The article "The Relationship between Ovarian Ultrasound Parameters and Endocrine and Metabolic Indicators in Patients with Ovarian Syndrome" was retracted in 2023. Reasons: unreliable results or conclusions; concerns about the data; concerns about the peer review; concerns about the citations.

# The Relationship between Ovarian Ultrasound Parameters and Endocrine and Metabolic Indicators in Patients with Ovarian Syndrome

**DOI:** 10.1155/2022/7238344

**Published:** 2022-07-30

**Authors:** Changqing Sheng, Jin Zhang, Jiang Jue

**Affiliations:** ^1^Department of Ultrasound, Northwest Women's and Children's Hospital, Xi'an, Shaanxi 710061, China; ^2^Department of Ultrasound, The Ninth Hospital of Xi'an, Xi'an, Shaanxi, China; ^3^Department of Ultrasound, The Second Affiliated Hospital of Xi'an Jiaotong University, Xi'an, China

## Abstract

**Objective:**

The aim of this study is to investigate the relationship between the levels of endocrine and metabolic indicators and ovarian ultrasonography indicators in patients with ovarian syndrome (PCOS).

**Methods:**

Three hundred and forty patients with PCOS from January 2017 to February 2022 were selected as the observation group, and 340 healthy women of the same age were selected as the control group. A retrospective analysis was performed to observe the levels of endocrine and metabolic indicators and ovarian ultrasound examination indicators in the two groups.

**Results:**

The levels of testosterone, dehydroepiandrosterone (DHEA-S), luteinizing hormone (LH), LH/FSH, blood glucose, and insulin were higher in the observation group than those in the control group. The levels of low-density lipoprotein (LDL) and free insulin-like growth factor (IGF-I) were higher in the observation group than those in the control group. However, the level of high-density lipoprotein (HDL) was lower in the observation group than that in the control group. The ovarian interstitial area, total ovarian area, ovarian volume, number of follicles, uterine artery pulsatility index (PI), and resistance index (RI) were higher in the observation group than those in the control group. Pearson correlation analysis concluded that estrone (E1) levels in PCOS patients were correlated with ovarian interstitial area, total ovarian area, and ovarian volume. In addition, E1 levels correlated with LH levels, LH/FSH, testosterone, DHEA-S, and progesterone at *P* < 0.05. Compared with different treatment methods, the total testosterone, LH, and LH/FSH levels in the two groups were decreased compared with those before treatment, and the degree of decrease in the combined treatment group was more significant than that in the treatment alone group.

**Conclusion:**

The levels of endocrine metabolism and ovarian ultrasound in PCOS patients are abnormal and there is a close relationship between the levels of endocrine metabolism and ovarian ultrasound. Attention should be paid to the monitoring and regulation of endocrine metabolism and ovarian ultrasound. Integrated traditional Chinese and western medicine can greatly improve the hormone levels in PCOS patients.

## 1. Introduction

Polycystic ovary syndrome (PCOS) is one of the most common endocrine disorders in women of childbearing age and mostly occurs in women aged 20–40 in childbearing periods. Its prevalence is between 5% and 10% [1]. The causes of PCOS include genetic factors, environmental factors, or obesity. PCOS is an ovarian dysfunction syndrome characterized by hyperandrogenism and ovarian morphology [2]. Associated symptoms and signs may include hyperinsulinemia, insulin resistance, dyslipidemia, dysfunctional uterine bleeding, endometrial cancer, hypertension, cardiovascular disease, and infertility [3–5]. Partial women with PCOS exhibit hirsutism, acne, obesity, and acanthosis nigricans as common associated features [6, 7].

It also involves abnormal secretion of gonadotropins, such as elevated LH levels, and a subsequent increase in the LH to follicle stimulating hormone (FSH) ratio in addition to elevated androgen levels [1] in endocrine and metabolic aspects, which are thought to be common features of PCOS [8, 9]. Elevated levels of anti-Samuel's canal hormone (AMH) are another typical feature [10]. Serum AMH levels are higher in PCOS patients than healthy controls and positively correlated with follicle count [11, 12]. *E*1, estradiol (*E*2), and estriol (*E*3) are endogenous estrogens [13]. A common hormonal feature in PCOS patients is elevated serum *E*1 levels and subsequent elevated *E*1/*E*2 ratios [14].

The consensus on PCOS criteria includes sonographic ovarian morphology as a relevant marker [15]. However, it is uncertain whether ovarian morphological parameters can predict the degree of PCOS and the response to treatment [16]. Among previous studies examining the association between ultrasound and clinical indicators, positive associations have been noted between androgens, gonadotropins, and menstrual cycle length and follicle count, ovarian interstitial area, and ovarian volume [17, 18]. It has been reported that there is a positive correlation between follicle number, ovarian volume, and insulin resistance markers [19]. However, other studies did not find this positive or opposite association [20, 21]. This study aimed to clarify the relationship between clinical, hormonal metabolic, and ultrasonographic features of PCOS using well-defined PCOS population, reliable ultrasonographic parameters.

## 2. Materials and Methods

### 2.1. Study Design and Participants

Three hundred and forty patients with PCOS from January 2017 to February 2022 were selected as the observation group and three hundred and forty patients healthy women of the same age who were treated during the same period were selected as the control group for retrospective analysis. The patients were from Northwest Women's and Children's Hospital and the Second Affiliated Hospital of Xi'an Jiaotong University. The patients in the observation group were 27.0 ± 2.5 years old on average (range 18 to 36) and the average BMI value was 22.7 ± 1.6 kg/m^2^ (range 18.4 to 26.6). The patients in the control group were 27.2 ± 2.9 years on average (range 19 to 37) and the average BMI value was 22.9 ± 1.2 kg/m^2^ (range 18.4 to 26.6). There was no difference in baseline data of patients in the two groups (*P* > 0.05). Informed consent was obtained from all patients. Endocrine levels and ovarian ultrasound parameters were completed in both groups. First, fasting venous blood samples were collected from both groups (patients with PCOS were sampled at about 2–5 days of menstruation). The blood samples were centrifuged at a centrifugation time of 5.0 min and a centrifugation rate of 3000 r/min. After centrifugation, the serum was taken for quantitative detection of endocrine and metabolic levels by an enzyme-linked immunosorbent assay. In addition, color doppler ultrasonography was performed. The above examinations and tests were completed by experienced professionals. All patients signed the informed consent, and the study was approved by the Ethics Committee (No. NH201-12).

### 2.2. Observation Indicators

The quantitative detection of endocrine and metabolic levels mainly includes testosterone, dehydroepiandrosterone, LH, FSH, LH/FSH, androstenedione, AMH, PRL, progesterone, blood glucose, blood lipid, IGF-I, insulin-like growth factor binding protein-1 (IGFBP-1), insulin, serum *E*1, *E*2, and other indicators. Ovarian ultrasound parameters mainly include ovarian interstitial area (SA) and total ovarian area (TA), ovarian volume (V), number of follicles (FN), uterine artery PI and RI, ovarian interstitial artery PI, and RI and other indicators; Pearson correlation was used to analyze the relationship between serum *E*1 levels and clinical, ultrasound, and endocrine and metabolic index levels.

PCOS patients were randomly divided into two groups: integrated traditional Chinese and western medicine combined treatment group (170 cases) and western medicine single treatment group (170 cases).

Traditional Chinese medicine treatment formula: Radix Bupleuri, Radix Paeoniae Rubra, Radix Paeoniae Alba, Radix Zelan, Herba Leonuri, Radix Liu Shunu, Radix Puhuang, Radix Achyranthis Bidentatae, Semen Cuscutae, Fructus Lycii, Cistanche deserticola, Curculigo, Epimedium, and Caulis Spatholobi.

### 2.3. Inclusion and Exclusion Criteria

The inclusion criteria were as follows: (1) PCOS patients who meet the diagnostic criteria by ultrasound and endocrine examination. (2) Age ≥ 18 years.

The exclusion criteria were as follows: (1) Patients with previous endocrine diseases such as hyperprolactinemia, thyroid disease, congenital adrenocortical hyperplasia, and Cushing's syndrome; (2) allergy to the traditional Chinese medicine used in the experiment; (3) combined with severe liver and kidney, cardiovascular and reproductive system diseases; and (4) psychiatric history, unable to cooperate with the examiner;

### 2.4. Statistical Analysis

SPSS 26.0 statistical software was used to analyze the data. The clinical data (measurement data) were expressed as mean ± standard deviation (*x* ± *S*). One-way ANOVA was used for comparison between groups. The *t*-test was used for intragroup comparison, the analysis of variance was used for the comparison between groups, and the Pearson correlation analysis was used for correlation. *P* < 0.05 was considered to be statistically significant.

## 3. Results

### 3.1. Comparison of Hormone and Blood Glucose Levels

There was no significant difference in the levels of diketone, FSH, PRL, and progesterone between the two groups (*P* > 0.05); however, the levels of total testosterone, free testosterone, dehydroepiandrosterone, LH, LH/FSH, blood glucose, and insulin in the observation group were significantly higher than those of the control group (*P* < 0.05). See details in Table 1.

### 3.2. Comparison of Blood Lipid and IGF Levels

There was no significant difference in total cholesterol, triglyceride, IGF-I, and IGFBP-1 levels between the two groups (*P* > 0.05); however, the LDL and free IGF-I levels in the observation group were significantly higher than those of the control group (*P* < 0.05). The HDL level of the observation group was significantly lower than that of the control group (*P* < 0.05). See details in Table 2.

### 3.3. Comparison of Ultrasound Parameters

As shown in Table 3, the ovarian interstitial area (SA), total ovarian area (TA), ovarian volume (V), number of follicles (FN), PI, and RI of the uterine artery in the observation group were higher than those of the control group (*P* < 0.05), and the PI and RI of ovarian interstitial artery were lower than the control group (*P* < 0.05).

### 3.4. Correlation Analysis between Serum E1 Level and Clinical, Ultrasound, and Endocrine and Metabolic Parameters in PCOS Patients

As shown in Table 4, E1 levels were significantly correlated with SA, TA, and V (*P* < 0.05). There was no significant correlation between the *E*1 level and age, BMI index (*P* > 0.05). In the analysis of the relationship between *E*1 level and other hormone indicators, the *E*1 level was significantly correlated with serum LH level, LH/FSH, total testosterone, free testosterone, DHEA-S, and progesterone (*P* < 0.05). There was a significant correlation between the *E*1/*E*2 ratio and free testosterone level (*P* < 0.05).

### 3.5. Comparison of Endocrine Parameters after Different Treatment Methods

The PCOS patients in the observation group were equally divided into two groups, one group was given combined treatment and the other group was given alone treatment. After treatment, total testosterone, LH, and LH/FSH levels in both groups were lower than before (*P* < 0.05). The degree of reduction in the combined treatment group was more significant than the single treatment group (*P* < 0.05). See details in Table 5.

## 4. Discussion

The endocrine and metabolic status of PCOS patients are relatively abnormal, which leads to important causes of abnormal uterine bleeding, infertility, and other adverse conditions, so the treatment needs of women in gestational age are often high [22]. This study aimed to investigate the relationship between the levels of endocrine and metabolic indicators and ultrasound parameters in PCOS patients. The results showed that the levels of total testosterone, free testosterone, dehydroepiandrosterone, LH, LH/FSH, blood glucose, and insulin in the PCOS group were significantly higher than those in the control group. Increased LH secretion leads to increased androgen production by theca cells, and increased conversion of androgens in theca cells leads to increased production of androstenedione, which is also an important cause of hirsutism and acne in PCOS patients [1, 11, 23]. It is also well-known that PCOS patients will develop insulin resistance, which is not difficult to explain the manifestations of increased blood glucose in patients [24]. This study also concluded that PCOS LDL and free IGF-I levels were significantly higher and HDL levels were significantly lower in the observation group than in the control group. Previous studies have found that among women with PCOS, obesity tends to be associated with a more atherosclerotic lipid profile [14, 25]. Some scholars have shown that women with PCOS disease will develop carotid atherosclerosis earlier, which has nothing to do with the women's body mass index. Obese adolescents with PCOS have higher low-density lipoprotein and lower high-density lipoprotein levels compared with nonobese adolescents [26]. The dysregulation of the IGF system has been implicated in the pathophysiology of PCOS. IGF-1 and insulin have been shown to stimulate proliferation of theca interstitial cells and enhance LH-stimulated androgen synthesis in these cells. It has been suggested that hyperandrogenism and increased peripheral androgen turnover in PCOS patients may be mediated by free IGF-I [27].

The ovarian SA, TA, V, FN, PI, and RI of uterine artery were higher than those of the control group, and the PI and RI of ovarian interstitial artery were lower than that of the control group (*P* < 0.05). Increased number of follicles and ovarian volume are two main features of ultrasonography in women with PCOS [28]. Elevated *E*1 levels and subsequent increased *E*1/*E*2 ratio are well-known hormonal characteristics in PCOS patients, but studies on the relationship between *E*1 levels and other basic characteristics in PCOS patients are lacking. In this study, we found that serum *E*1 levels were not only associated with LH and androgen levels but also with ultrasound volume parameters. As mentioned earlier, increased LH secretion in PCOS patients leads to increased metandienone, which can be converted to *E*1 by aromatase. These pathophysiological mechanisms may explain why there was a strong correlation between *E*1 levels and LH and androgen levels in this study. In addition, it has been found that there is a very significant relationship between follicle count and ovarian volume and serum AMH and LH levels. Needless to say, ovarian morphology is an essential feature of PCOS, which is an important diagnostic criterion [29]. Lack of ultrasound data may lead to missed diagnosis of PCOS patients. Ideally, transvaginal ultrasound should be performed to optimize image resolution, particularly in obese patients [30]. For patients who are unable to undergo vaginal ultrasonography, the levels of endocrine and metabolic indicators will also provide many useful information, and the combination of the two groups plays an important role in the diagnosis or follow-up of PCOS patients [31]. After different treatment methods, after treatment, the total testosterone, LH, and LH/FSH levels in both groups were lower than before. The degree of reduction in the combined treatment group was more significant than that in the treatment alone group. These results indicate that integrated traditional Chinese and western medicine treatment can greatly improve hormone levels in PCOS patients. At present, traditional Chinese medicine is a common method to treat polycystic ovarian cysts and can regulate women's general conditions. Previous studies have also shown that integrated traditional Chinese and western medicine treatment improves the therapeutic efficacy of PCOS patients, improves the hormone levels and symptoms of patients, and brings a new direction for the treatment of PCOS patients.

In summary, the endocrine and metabolic levels and ovarian ultrasound detection indicators in PCOS patients showed an abnormal state, and the endocrine and metabolic levels were closely related to ovarian ultrasound detection indicators. In clinical aspects, attention should be paid to the monitoring of endocrine and metabolic levels and ovarian ultrasound detection indicators in PCOS patients, and integrated traditional Chinese and western medicine treatment can greatly improve the hormone levels in PCOS patients.

## Figures and Tables

**Table 1:** Comparison of hormone and blood glucose levels between the two groups.

	Observation group (*N* = 340)	Control group (*N* = 340)
Total testosterone (ng/ml)	0.62 ± 0.22^a^	0.53 ± 0.38
Free testosterone (pg/ml)	0.72 ± 0.84^a^	0.64 ± 0.69
Androstenedione (ng/mL)	3.41 ± 0.75	3.39 ± 0.97
Dehydroepiandrosterone (UG/DL)	202.39 ± 107.70^a^	191.18 ± 104.51
FSH (IU/L)	6.09 ± 0.28	6.11 ± 0.29
LH (IU/L)	12.62 ± 5.40^a^	9.18 ± 4.73
LH/FSH	2.93 ± 0.71^a^	1.21 ± 1.03
PRL (ng/ml)	18.25 ± 8.06	18.01 ± 7.96
Progesterone (ng/ml)	1.14 ± 0.51	1.09 ± 0.72
Glucose (mg/dL)	89.74 ± 13.77^a^	86.03 ± 12.90
Insulin (uU/mL)	22.35 ± 10.02^a^	18.56 ± 9.71

Compared with the control group, a represents *P* < 0.05.

**Table 2:** Comparison of lipid and IGF levels between the two groups.

Group	*n*	Total cholesterol (mg/dL)	Triglyceride (mg/dL)	LDL (mg/dl)	HDL (mg/dl)	IGF-I (ng/ml)	IGFBP-1 (ng/ml)	Free IGF -I (ng/ml)
Observation group	340	154.39 ± 10.36	86.35 ± 42.71	101.58 ± 23.26	40.60 ± 9.35	403.02 ± 129.73	0.92 ± 1.63	8.13 ± 3.34
Control group	340	153.57 ± 19.82	85.35 ± 44.48	86.80 ± 16.98	51.20 ± 10.29	395.56 ± 137.60	1.13 ± 2.17	6.51 ± 4.27
*t*		0.676	0.299	9.463	14.058	0.727	1.427	5.510
*P*		0.499	0.765	<0.001	<0.001	0.467	0.154	<0.001

**Table 3:** Comparison of ultrasonic indexes between the two groups.

Group	*n*	SA (cm^2^)	TA (cm^2^)	V (ml)	FN (number)	Ovarian interstitial artery PI	Ovarian interstitial artery RI	Uterine artery PI	Uterine artery RI
Observation group	340	1.04 ± 0.32	5.42 ± 0.79	13.13 ± 2.32	13.27 ± 5.66	0.88 ± 0.12	0.49 ± 0.02	2.02 ± 0.12	0.82 ± 0.07
Control group	340	0.99 ± 0.13	4.77 ± 0.60	12.37 ± 1.94	10.93 ± 2.96	0.91 ± 0.15	0.51 ± 0.04	1.95 ± 0.03	0.79 ± 0.06
*t*		2.669	12.082	4.634	6.755	2.88	8.246	10.435	6.000
*P*		0.008	<0.001	<0.001	<0.001	0.004	<0.001	<0.001	<0.001

**Table 4:** Correlation analysis of serum *E*1 level with clinical, ultrasonic, and endocrine and metabolic indicators.

	*E*1		*E*2		*E*1/E2	
	*r*	*P*	*r*	*P*	*r*	*P*
Age (years)	−0.030	0.720	0.053	0.076	−0.009	0.785
BMI (kg/m^2^)	0.043	0.319	−0.066	0.530	0.127	0.320
SA (cm^2^)	0.237	**<0.001**	−0.359	0.249	0.206	0.351
TA (cm^2^)	0.429	**<0.001**	−0.234	0.655	0.007	0.734
V (ml)	0.509	**<0.001**	0.353	0.154	0.093	0.511
FN (number)	0.322	0.870	0.076	0.246	0.087	0.722
Interstitial ovarian artery PI	0.410	0.625	0.091	0.499	0.055	0.403
Ovarian interstitial artery RI	0.352	0.179	0.085	0.765	0.098	0.472
Uterine artery PI	0.465	0.058	0.117	0.344	0.192	0.239
Uterine artery RI	0.399	0.112	0.125	0.143	0.155	0.332
AMH (ng/ml)	0.308	0.275	−0.099	0.784	0.075	0.616
FSH (IU/L)	−0.44	0.344	−0.367	0.896	−0.005	0.180
LH (IU/L)	0.229	**<0.001**	0.149	0.673	−0.037	0.110
LH/FSH	0.351	**<0.001**	0.074	0.157	−0.007	0.050
Total testosterone (ng/ml)	0.317	**<0.001**	−0.065	0.534	0.818	0.935
Free testosterone (pg/ml)	0.288	**<0.001**	−0.097	0.314	0.515	**0.002**
Dehydroepiandrosterone (UG/DL)	0.381	**0.039**	−0.116	0.376	0.076	0.989
Progesterone (ng/ml)	0.230	**<0.001**	0.173	0.415	−0.037	0.434

**Table 5:** Comparison of endocrine indexes after different treatment methods.

Group	*n*	Total testosterone (ng/ml)		LH (IU/L)		LH/FSH	
		Before treatment	After treatment	Before treatment	After treatment	Before treatment	After treatment
Combination therapy group	170	0.62 ± 0.22	0.53 ± 0.26^a^	12.62 ± 5.40	10.27 ± 3.66^a^	2.93 ± 0.71	1.31 ± 0.42^a^
Treatment group	170	0.62 ± 0.22	0.60 ± 0.19^a^	12.62 ± 5.40	12.03 ± 4.96^a^	2.93 ± 0.71	2.23 ± 0.74^a^
*t*		—	2.834	—	3.723	—	14.098
*P*		—	0.005	—	<0.001	—	<0.001

## Data Availability

The data used to support the findings of this study are available from the corresponding author upon request.
